The article "Activation of CD137 Signaling Enhances Vascular Calcification through c-Jun N-Terminal Kinase-Dependent Disruption of Autophagic Flux" was retracted in 2022. Reason: duplicated images.

# Activation of CD137 Signaling Enhances Vascular Calcification through c-Jun N-Terminal Kinase-Dependent Disruption of Autophagic Flux

**DOI:** 10.1155/2018/8407137

**Published:** 2018-09-26

**Authors:** Rui Chen, Yao Xu, Wei Zhong, Bo Li, Ping Yang, Zhong Qun Wang, Chen Shao, Cui Ping Wang, Jin Chuan Yan

**Affiliations:** Department of Cardiology, Affiliated Hospital of Jiangsu University, Zhenjiang, Jiangsu Province, China

## Abstract

**Background:**

Vascular calcification is widespread and clinically significant, contributing to substantial morbidity and mortality. Calcifying vascular cells are partly derived from local vascular smooth muscle cells (VSMCs), which can undergo chondrogenic or osteogenic differentiation under inflammatory environment. Recently, we have found activation of CD137 signaling accelerated vascular calcification. However, the underlying mechanism remains unknown. This study aims to identify key mediators involved in CD137 signaling-induced vascular calcification in vivo and in vitro.

**Methods:**

Autophagy flux was measured through mRFP-GFP-LC3 adenovirus and transmission electron microscopy. Von Kossa assay and alkaline phosphatase (ALP) activity were used to observe calcification in vivo and in vitro, respectively. Autophagosome-containing vesicles were collected and identified by flow cytometry and Western blot. Autophagy or calcification-associated targets were measured by Western blot, quantitative real-time PCR, and immunohistochemistry.

**Results:**

Treatment with the agonist-CD137 displayed c-Jun N-terminal kinase- (JNK-) dependent increase in the expression of various markers of autophagy and the number of autophagosomes relative to the control group. Autophagy flux experiments suggested that agonist-CD137 blocked the fusion of autophagosomes with lysosomes in cultured VSMCs. Calcium deposition, ALP activity, and the expression of calcification-associated proteins also increased in agonist-CD137 group compared with anti-CD137 group, which could be recovered by autophagy stimulator rapamycin. Autophagosome-containing vesicles collected from agonist-CD137 VSMCs supernatant promoted VSMC calcification.

**Conclusion:**

The present study identified a new pathway in which CD137 promotes VSMC calcification through the activation of JNK signaling, subsequently leading to the disruption of autophagic flux, which is responsible for CD137-induced acceleration of vascular calcification.

## 1. Introduction

Vascular calcification is preceded by vascular smooth muscle cell (VSMC) adaptation and dysfunction, which ultimately leads to the initiation of active osteogenic process within the vessel wall [1]. Vascular calcification is a common complication in patients with diabetes and atherosclerosis and is a major risk factor for cardiovascular morbidity and mortality [2, 3]. Inflammation plays a major role in VSMC osteogenic transdifferentiation [4] and vascular calcification [5–7].

The article "Activation of CD137 Signaling Enhances Vascular Calcification through c-Jun N-Terminal Kinase-Dependent Disruption of Autophagic Flux" was retracted in 2022. Reason: duplicated images.

CD137, a member of the tumor necrosis factor receptor superfamily (TNFRSF), is expressed in a variety of immune cells and is involved in autoimmunine and inflammatory reactions [8]. The expression of CD137 can also be induced in VSMCs and endothelial cells (ECs) under proinflammatory conditions [9]. Both CD137 and CD137 ligands are found in human atherosclerotic lesions, and their expression increases with plaque progression [10]. Deficiency of CD137 reduces atherosclerosis in mice on both chow and high-fat diets [11]. In addition, we recently showed CD137 signaling contributed to the calcification of atherosclerotic lesions [12]. However, the underlying mechanisms whereby CD137 signaling affects vascular calcification remain largely unknown.

Autophagy is a highly conserved process by which unnecessary or damaged cellular components are degraded by lysosomes [13]. Functional autophagy is necessary to maintain cardiovascular homeostasis [14]. In contrast, impaired autophagy contributes to a wide range of vascular pathologies including atherosclerosis and calcification [15, 16]. Reactive oxygen species production, oxidized lipoproteins, endoplasmic reticulum stress, and hypoxia are involved in triggering the process of autophagy in atherosclerotic plaques [17–19]. Interestingly, autophagy-associated inflammasomes contribute to atherosclerotic progression [20]. However, the mechanisms linking autophagy to inflammation and vascular calcification remain unclear. Here, we investigated the role of autophagy in CD137-mediated VSMC osteogenic transdifferentiation and vascular calcification.

## 2. Materials and Methods

### 2.1. Ethics Statement and Tissue Samples

All animal experimental procedures were conducted in accordance with institutional guidelines for the care and use of laboratory animals in Jiangsu University, Zhenjiang, China, and conformed to the National Institutes of Health Guide for Care and Use of Laboratory Animals (Publication No. 85-23, revised 1996). Male, six eight-week-old ApoE^−/−^ mice were purchased from Vital River Laboratories (Distributor of Jackson Laboratory, Beijing, China) and housed in pathogen-free standard conditions. The atherosclerotic plaque model was generated through Western diet (mainly consisted of 0.15% cholesterol, 20% fat, 49% carbohydrate, 17.3% protein, and 5% fiber) and divided into the following four groups (*n* = 6/group): control group, agonist-CD137 group, c-Jun N-terminal kinase (JNK) inhibition group, and DMSO group. Mice in control and agonist-CD137 group were injected with 200 *μ*g of isotype antibody (eBioscience) and mouse agonist-CD137 (R&D, USA) once per week, respectively. The mice were injected with 30 mg/kg of SP600125 (Cell Signaling Technology, American) followed by 200 *μ*g of mouse agonist-CD137 in JNK inhibition group. In order to exclude the effects of solvents, mice in control group were injected with equal amount of dimethylsulfoxide (DMSO). All reagents were injected intraperitoneally and once per week. The mice were euthanized through CO_2_ anesthesia after 10 weeks of treatment. Aortas were removed from identical sites in each mouse for future assays.

The article "Activation of CD137 Signaling Enhances Vascular Calcification through c-Jun N-Terminal Kinase-Dependent Disruption of Autophagic Flux" was retracted in 2022. Reason: duplicated images.

### 2.2. Extraction of Mouse Aortic Protein

The aortas obtained from mice in each groups were homogenized with 100 *μ*L RIPA Lysis Buffer. The homogenate was placed on ice for 1 h then centrifuged at 15000*g* for 15 minutes at 4°C. The supernatant was collected and denatured in boiling water for 8 min. The protein samples were stored at −20°C until further analysis.

### 2.3. Cell Culture

The VSMCs were isolated from the aorta of male, eight-week-old C57BL/6J mice as reported previously. Briefly, the thoracic aorta was dissected under a surgical microscope. The aorta was removed and washed with PBS several times before treated with type II collagenase. The vessels were then cut into pieces and cultivated in a humidified incubator containing 5% CO_2_ at 37°C to obtain VSMCs. Cells were seeded into six well plates and divided into four groups: control group, agonist-CD137 group, JNK inhibition group, and DMSO group. All groups were prestimulated with mixed cytokines (CM: 10 ng/ml interleukin 1-*β* (IL-1*β*), 10 ng/ml interferon- (IFN-) *γ*, and 10 ng/ml tumor necrosis factor-alpha (TNF-*α*)) for 24 h before treatment. Agonist-CD137 group was then treated with recombinant protein of agonist-CD137 (10 *μ*g/ml). JNK inhibition group was stimulated by SP600125 (10 *μ*M) for 30 minutes and then treated with agonist-CD137 (10 *μ*g/ml). Same amount of DMSO as JNK inhibition group was added to DMSO group. Chloroquine (CQ) (10 *μ*M) and rapamycin (500 nM) were used as autophagy inhibitor and stimulator, respectively.

### 2.4. Von Kossa Assay

Cells were cultured in calcification medium (DMEM + 10 mmol/L beta-glycerine phosphate + 10% fetal bovine serum (FBS) for 15 days and the medium were replaced every other days. VSMCs were fixed with 4% paraformaldehyde and incubated with 2% silver nitrate solution. The cells were then placed under ultraviolet light for 30 min. Uncombined silver was removed with 5% sodium thiosulfate for 5 min and stained with nuclear fast red for 3 min after washing with phosphate-buffered saline (PBS) 3 times. Images were obtained using an Olympus microscope.

The article "Activation of CD137 Signaling Enhances Vascular Calcification through c-Jun N-Terminal Kinase-Dependent Disruption of Autophagic Flux" was retracted in 2022. Reason: duplicated images.

### 2.5. mRFP-GFP-LC3 Adenovirus Puncta Assay

The autophagy flux was assessed by mRFP-GFP-microtubule-associated protein 1 light chain 3 (LC3) adenovirus probe assay. VSMCs were seeded into 12 well plate and transfected with 80 multiplicity of infection of mRFP-GFP- LC3 adenovirus (Han Heng, China) in serum-free medium. The medium was changed to complete medium after six hours followed by treatment with agonist-CD137 (10 *μ*g/ml) in the presence or absence of either DMSO or SP600125 (10 *μ*M). Cells were fixed with 4% paraformaldehyde and then stained with DAPI. Images were obtained using an Olympus microscope. The yellow and red punctum were calculated to observe autophagy flux.

### 2.6. Transmission Electron Microscopy

Cells were centrifuged at 500*g* for 5 min and washed three times. Cell samples and carotid section were fixed with cold 2.5% glutaraldehyde solution and sent to Nanjing Medical University (Nanjing, China) for detection. The random three horizons were selected to calculate the quantity of lysosomes and autophagosomes which represent the autophagy process.

### 2.7. Western Blot

Protein samples were extracted using a protein extraction reagent and separated by an SDS-PAGE polyacrylamide gel and transferred to PVDF membranes. The membranes were blocked and incubated with antibodies against Beclin1, SQSTM1/p62 (Abcam, USA), bone morphogenetic protein 2 (BMP-2), runt-related transcription factor 2 (Runx2), *β*-actin (Immunoway, USA), and LC3B antibody (CST, USA). After incubation with secondary antibodies, bands were detected by enzyme-linked chemiluminescence according to the manufacturer's protocol (ECL; Bio-Rad).

### 2.8. mRNA Extraction and Real-Time Quantitative PCR

Total RNAs were extracted from cells of each group and purified using the RNeasy Mini Kit per manufacturers' instructions. Reverse transcription was performed using Thermo Fisher RT reagents. Primers were synthesized by Sangon (Shanghai, China). AceQ qPCR SYBR Green Master Mix were bought from Vazyme (Nanjing, China).

### 2.9. O-Cresolphthalein Complexone and Alkaline Phosphatase Activity Assay

The content of extracellular calcium was measured by o-cresolphthalein complexone and alkaline phosphatase (ALP) activity (Nanjing Jiancheng Bioengineering Research Institute, China). Cell medium was collected and centrifuged to remove cell debris. The supernatant was harvested and buffer solution and matrix solution were added. After incubation and color development, the absorbance was measured at 520 nm with the microplate reader. The cells were washed by PBS for three times, 0.6 mmol/L diluted hydrochloric acid was used to dissolve the extracellular calcium. The o-cresolphthalein complexone was added into the suspension and measured at 575 nm. The activity values were calculated and normalized to the protein content.

The article "Activation of CD137 Signaling Enhances Vascular Calcification through c-Jun N-Terminal Kinase-Dependent Disruption of Autophagic Flux" was retracted in 2022. Reason: duplicated images.

### 2.10. Immunohistochemistry

Serial sections were stained using an immunohistochemistry kit (CW Biotech, China). The samples were incubated with antibodies against LC3B (1 : 300), Beclin1 (1 : 300), and p62 (1 : 300) at 4°C overnight. All assays were conducted according to the manufacturer's instructions. The integrated option density (IOD) value was measured using the Image-Pro Plus 6.0 software. Cells were disposed similar with animal study; BMP2 (1 : 100) was used to observe the osteoblast-like phenotype of VSMCs.

### 2.11. The Isolation of Autophagosome-Containing Vesicles

Autophagosome-containing vesicles were harvested from VSMCs in control group, agonist-CD137 group, and anti-CD137 group. The cells and the supernatant were harvested and spun at 480*g*. The acquired supernatant was spun at 12000*g* for 20 min to harvest the autophagosome-containing pellet [21]. The pellet was resuspended with PBS and protein concentration detected using BCA kit (Vazyme Biotech, Nanjing, China). Autophagosome-containing vesicles were added to VSMCs to induce calcification at the final concentration of 15 *μ*g/ml.

### 2.12. Flow Cytometry

Flow cytometry was performed to detect the LC3 level of autophagosome-containing vesicles. Vesicles were acquired and washed with PBS. Anti-LC3B-PE (eBioscience, USA) was diluted according to the protocol and was added to 100 *μ*l cell suspension for 30 min at 4°C. After the incubation, the cells were washed one time and then analyzed by flow cytometry (BD Canto II).

### 2.13. Statistical Analysis

Data are expressed as the mean ± SEM of at least three independent experiments (in vitro) and were compared by *t*-test or ANOVA using SPSS version 12.0 (SPSS, Chicago, IL, USA). *P* < 0.05 was considered significant.

## 3. Results

### 3.1. CD137 Signaling Activation Induced Calcification and Autophagy in ApoE^−/−^ Mice

The calcification of aorta was observed through Von Kossa staining. Compared to the control group, the lesion and calcification areas formed in vessels of agonist-CD137 group was significantly greater. In the anti-CD137 group, the plaque was attenuated and no obvious calcification areas existed in lesions. To determine whether calcification is associated with autophagy, we measured the levels of LC3B and Beclin1 through immunohistochemistry (Figures 1(a) and 1(b)). Consistent with the findings mentioned above, Western blot analysis showed that p62 and the ratio of LC3II/I also increased in agonist-CD137 group (Figure 1(c)) which suggests that the autophagy flux may be obstructed in CD137 signaling induced plaque formation. Moreover, the levels of calcification-associated proteins (BMP2, RUNX2) increased in agonist-CD137 group but decreased when CD137 signaling was blocked (Figure 1(d)). The result of transmission electron microscopy revealed that the quantity of autophagosome increased in agonist-CD137 group, suggesting the accumulation of autophagosome (Figure 1(e)).

The article "Activation of CD137 Signaling Enhances Vascular Calcification through c-Jun N-Terminal Kinase-Dependent Disruption of Autophagic Flux" was retracted in 2022. Reason: duplicated images.

### 3.2. CD137 Signaling Induced VSMC Autophagy and Calcification

VSMCs are the major component of vascular media and have been proved to play an important role in calcification. We examined the expression of autophagic markers in VSMCs in vitro. It showed that agonist-CD137 increased the ratio of LC3II/LC3I and reached the peak at 10 *μ*g/ml. Furthermore, the increased ratio was the greatest at 6 h after treatment of 10 *μ*g/ml recombinant protein (Figure 2(a)). To determine the increase in the ratio of LC3II/LC3I correlated with the autophagy induction or a block in autophagosome clearance, we repeated the experiment in the absence or presence of CQ, an inhibitor of autophagosome-lysosome fusion. CQ treatment further elevated the ratio of LC3II/LC3I and the autophagy substrate p62 under agonist-CD137 (Figure 2(b)). To determine whether CD137 signaling induced the blockage of autophagy flux, VSMCs were transfected with mRFP-GFP-LC3 adenovirus for 6 h. The number of yellow fluorescent in agonist-CD137 group increased compared to control and anti-CD137 group while the red fluorescent declined in agonist-CD137 group (Figure 2(c)). The results suggest that CD137 signaling induces autophagy dysfunction in VSMCs.

We then investigated if the autophagy dysregulation is the mediator of the CD137 signaling-mediated increase in VSMC calcification by pretreating the cells with autophagy stimulator rapamycin. The mRNA and protein levels of calcification-associated protein BMP2 and Runx2 increased in agonist-CD137 group compared to control group and anti-CD137 group (Figures 3(a) and 3(c)), which is consistent with the results from Von Kossa assay (Figure 3(e)). The ALP activity assay and calcium deposition also showed the increment in agonist-CD137 group (Figure 3(d)). However, as observed in Figure 3, the agonist-CD137 treated cells in the presence of rapamycin showed significantly decreased expression of BMP2 and Runx2, the lower ALP activity and calcium deposition.

### 3.3. JNK Pathway Is Involved in CD137-Induced Autophagy Dysfunction

As one of the important downstream targets of CD137 signaling, we evaluated the role of JNK pathway in CD137-induced autophagy. SP600125 was used to block JNK pathway in ApoE^−/−^ mice. Immunohistochemistry results showed that autophagy-associated proteins LC3B or p62 were increased in plaques induced by agonist-CD137, which could be rescued by SP600125 (Figures 4(a) and 4(b)). Western blot analysis of the tissues showed the same tendency (Figure 4(c)).

The article "Activation of CD137 Signaling Enhances Vascular Calcification through c-Jun N-Terminal Kinase-Dependent Disruption of Autophagic Flux" was retracted in 2022. Reason: duplicated images.

We then studied the association of JNK pathway and the expression of p62 and LC3 in VSMCs and found that CD137 activation elevated phosphorylated JNK. Inhibition of JNK through SP600125 caused reduced expression of p62 and LC3 compared to agonist-CD137 group (Figure 4(d)). The mRFP-GFP-LC3 adenovirus puncta assay revealed a brighter GFP fluorescence in agonist-CD137 group than control and anti-CD137 groups which means a dysfunction autophagy flux (Figures 4(e) and 4(f)). Results from transmission electron microscopy showed the quantity of autophagosome was increased after agonist-CD137 treatment, which was rescued by JNK blockage (Figures 4(g) and 4(h)).

### 3.4. The Secretion of Autophagosome-Containing Vesicles Induced by CD137 Promotes VSMC Calcification

To confirm that CD137 signaling induced the autophagy dysfunction and caused the accumulation of autophagosome, we asked whether the autophagosome can be secreted from VSMCs and led to the calcification. The vesicles in agonist-CD137 group was collected and identified by expression of LC3 through flow cytometry and Western blot (Figures 5(a) and 5(b)). BCA protein assay suggested that CD137 signaling activation may increase the autophagosome-containing vesicle production (Figure 5(c)) and autophagosome-containing vesicles derived from agonist-CD137 treated VSMCs exhibited more calcification than control as shown by Von Kossa assay, BMP2 staining (Figure 5(d)) and increased expression of BMP2 and Runx2 (Figure 5(e)).

## 4. Discussion

CD137 signaling is an important therapeutic target for development of vascular calcification [12]. Here, we have demonstrated for the first time that the activation of CD137 signaling could upregulate JNK phosphorylation which subsequently impaired the development of autophagic flux and ultimately leading to the vascular calcification.

We found that activation of CD137 signaling with agonist-CD137 antibody increased the initiation of vascular autophagy but impaired the autophagic flux as evidenced by increased expression of LC3B, Beclin-1, and p62 in atherosclerotic lesions. Additionally, our in vivo data were supported by the in vitro observation that activation of CD137 signaling also induced the increment of LC3II/LC3Iratio and p62 expression in VSMCs. Autophagy is a dynamic process including nucleation, autophagosome formation, autophagosome-lysosome fusion, and lysosomal degradation [22]. Beclin-1 is accumulated at the early steps and forms a complex with class III phosphatidylinositol-4,5-bisphosphate 3-kinase which is responsible for autophagic vesicle nucleation [23]. LC3 consists of a soluble form LC3I and a lipidated form LC3II and has three isoforms LC3A, LC3B and LC3C in mammalian cells. During autophagy, the cytosolic proteolytically processed form LC3-I is conjugated to form LC3-phosphatidylethanolamine, LC3-II, which is recruited to the autophagosomal membrane [24]. Therefore, the increased ratio of LC3II/LC3I can be used as indicator of either upregulation of autophagosome synthesis or downregulation of autophagosome degradation [25]. There are no ideal techniques for assessing autophagic flux in vivo [26]. However, p62/SQDTM, a chaperone that shuttles intracellular protein aggregates into autophagosomes for degradation, has emerged as a useful marker of autophagic status since the entire p62/SQDTM1 protein aggregated complex is degraded after engulfment by the autolysosome. p62/SQDTM1 level is inversely correlated with autophagic flux [27]. Therefore, the combination of elevated Beclin-1, LC3B, and p62 which were observed in the vascular samples from mice treated with agonist-CD137 antibody indicates the accumulation of autophagy induction and the dysregulation of autophagy. Additional evidence linking autophagy and CD137 signaling by electron microscopic analysis revealed the accumulation of autophagosome after agonist-CD137 treatment. Furthermore, significant decrease in red puncta and increase in the number of yellow fluorescent in agonist-CD137 group showed the disruption of the autophagic flux, resulting from inhibition of autophagosome-lysosomal fusion. We also used CQ in VSMCs to obtain additional evidence for identifying autophagy as the downstream of CD137 signaling. It showed more increased expression of p62 and the ratio of LC3II/I when CQ combined with agonist-CD137, suggesting they have the similar effects on autophagy in VSMCs. Taken together, these data suggest that the dysfunctional autophagy induced by the activation of CD137 signaling is mainly due to defective autophagosome-lysosome fusion and impaired autophagic flux.

The article "Activation of CD137 Signaling Enhances Vascular Calcification through c-Jun N-Terminal Kinase-Dependent Disruption of Autophagic Flux" was retracted in 2022. Reason: duplicated images.

CD137 signaling has been shown to regulate JNK pathway in T cells [28], macrophage [29], and non-small-cell lung cancer cell [30]. JNK is a family of structurally similar serine-1 threonine kinase and its activity is barely detectable in the normal vascular but highly inducible when vascular cells are under inflammatory environment [31, 32]. Here, we demonstrated that phosphorylated JNK expression was increased after agonist-CD137 treatment in mouse aortas and VSMCs. It was shown that JNK signaling pathway plays an important role in various forms of autophagy [33, 34]. Xu et al. recently found that JNK inhibited autophagy in neurons by suppressing the expression of autophagy-related genes [35]. We demonstrated in the present study that inhibition of JNK by its inhibitor SP600125 reduced the expression of LC3II and p62 in vivo. Our in vitro studies showed that the dysfunction of autophagy flux can be rescued by JNK blockage in VSMCs as indicated by decreased quantity of autophagosome and GFP fluorescent after suppression of JNK by SP600125. These results suggest an essential role of JNK activation in mediating CD137 signaling-induced autophagy dysfunction. On the contrary, Haberzettl et al. found JNK activation is required for autophagy in rat VSMCs [36]. Jia et al. also revealed autophagy gene beclin1 expression could be induced by TNF-*α* through JNK pathway in plaque VSMCs [37]. These discrepancies suggest that the role of JNK autophagy is both context and cell type dependent. However, our data could not rule out the possibility that other mitogen-activated protein kinases are involved. Additional studies are warranted to dissect the precise signaling cascades that are responsible for disruption of autophagic flux by CD137 signaling in VSMCs.

Vascular calcification frequently occurs in the pathophysiological process of human arteries that is closely associated with coronary atherosclerosis [38]. Therefore, clarifying the underlying mechanisms involved in the initiation and development of calcification is important. Vascular calcification has been recognized as a dynamic and actively regulated process influenced by various factors, including inflammatory molecules [5].

The relationship between CD137 signaling and atherosclerosis has been proved in acute coronary syndrome patients, where both increased circulating CD137 levels and expression of CD137 on peripheral monocytes have been documented [39, 40]. More importantly, CD137 has been found in atherosclerotic plaques from patients and promoted lesion formation [10]. Recently, we found that CD137 signaling induced significant formation of atherosclerotic plaque calcification [12]. The main feature of vascular calcification is the osteogenic phenotype of the cells. VSMCs play a key role in vascular calcification [41]. The activation of CD137 signaling also induced VSMC calcification by upregulating the levels of BMP2 and Runx2 and increasing ALP activity and vice versa.

Although CD137 signaling has been demonstrated to promote calcification, the underlying mechanisms are still unclear. Given our findings of increased autophagy-related gene expression including beclin-1, LC3B, and p62 from plaque tissue, our data point to autophagy dysfunction as the key mechanism underlying CD137 induced activation of osteogenic program in VSMCs. The activation of CD137 signaling in VSMCs induces autophagy and impairs autophagic flux leading to the accumulation of autophagosomes in the cytoplasmic and secretion of vesicles. These vesicles were identified as LC3-positive compartment through flow cytometry and Western blot. LC3-postive structures include double-membrane autophagosome, autophagosome-like structure, noncanonical LC3 lipidation, and LC3-associated phagocytosis [42]. More studies need to investigate the nature of these autophagosome-containing vesicles. We further investigated whether autophagy functionally contributed to CD137 signaling-induced calcification. VSMCs are more prone to osteogenic/chondrogenic conversion stimulated by autophagosome-containing vesicles. Although how these autophagosome-containing vesicles affect VSMCs calcification remains unknown, some evidence suggest that inflammation may be involved in VSMC phenotypic transition through the loss of contractile markers followed by releasing the potent calcification promoting factor such as BMP2 from VSMCs [43]. BMP2 regulates osteoblast differentiation and bone formation through the induction of osteogenic transcription factor such as Runx2 [44]. Runx2 regulates the transcription of genes associated with osteoblast differentiation [45]. We also used the autophagy stimulator rapamycin obtaining additional evidence for identifying dysregulation of autophagy as a mediator involved in CD137 signaling-induced VSMC calcification. Our results suggested that the increased VSMC calcification in response to CD137 signaling may be induced primarily via autophagy dysregulation. The role of autophagic flux in maintaining normal vessel wall biology has been increasingly recognized, and autophagic dysregulation may be a common pathway implicated in atherosclerotic process [46]. Autophagy acts as an endogenous mechanism protecting against phosphorus-induced vascular calcification by reducing matrix vesicle release [47]. In line with previous reports, our data demonstrated that disruption of autophagy in response to CD137 signaling could promote the development of the osteochondrogenic VSMC phenotype. In contrast, Chiu et al. reported that autophagy was required for the osteogenic differentiation of mesenchymal stem cells [48]. This is not surprising as autophagy has dual roles in the development of atherosclerosis. It might differentially regulate osteogenic differentiation depending on cellular environment and disease status.

The article "Activation of CD137 Signaling Enhances Vascular Calcification through c-Jun N-Terminal Kinase-Dependent Disruption of Autophagic Flux" was retracted in 2022. Reason: duplicated images.

## 5. Conclusions

In summary, CD137 signaling-mediated phosphorylation of JNK plays an important role in mediating disruption of autophagic flux, resulting in VSMC osteogenic differentiation and acceleration of vascular calcification. Our study shed new light into the CD137-JNK-autophagic pathway, which paves the way to the development of novel therapeutic approach to treat vascular calcification.

## Figures and Tables

**Figure 1:** CD137 signaling activation induced calcification and autophagy in ApoE^−/−^ mice. (a, b) Von Kossa staining of calcification region and immunohistochemistry staining of Beclin1, LC3B, and p62 in the aorta of ApoE^−/−^ mice. (c, d) The expression of LC3, p62, and calcification-associated proteins (BMP2, RUNX2) in the aorta of ApoE^−/−^ mice was detected by Western blot. (e) Transmission electron microscopy was used to trace autophagosomes in aortic plaque of ApoE^−/−^ mice (red arrow: autophagosomes; black arrow: calcium deposition). Data are expressed as the mean ± SEM of at least three independent experiments. ^∗^ refers to *P* < 0.05; ^∗∗^ refers to *P* < 0.01.

**Figure 2:** CD137 signaling induced VSMC autophagy. (a) Primary mouse aortic VSMCs were stimulated by recombinant protein of agonist-CD137 (10 *μ*g/ml) for different concentrations and time. Western blot was applied to measure the expression of LC3B after treatment. (b) VSMCs were treated with CQ (10 *μ*mol/L) 15 min before agonist-CD137 treatment for 6 h followed by protein extraction for Western blot analyses of p62 and LC3B. (c) Image showing LC3B staining in each group of VSMCs infected with mRFP-GFP-LC3 adenovirus for 6 h. Data are expressed as the mean ± SEM of at least three independent experiments. ^∗^ refers to *P* < 0.05; ^∗∗^ refers to *P* < 0.01.

**Figure 3:** Preincubation with autophagy stimulator rapamycin attenuated CD137 signaling induced VSMCs calcification. (a–c) The protein and mRNA levels of BMP2 and Runx2 were analyzed by Western blot and RT-PCR, respectively. (d) Image showing extracellular ALP activity and calcium deposition in each group. (e) Von Kossa staining was applied to detect the calcification in VSMCs of each group. Data are expressed as the mean ± SEM of at least three independent experiments.^∗^ refers to *P* < 0.05; ^∗∗^ refers to *P* < 0.01.

**Figure 4:** JNK pathway was involved in autophagy dysfunction induced by CD137 signaling. (a–c) The expression of p-JNK, LC3B, and p62 in aortic plaque of ApoE^−/−^ was evaluated by immunohistochemistry staining and Western blot. (d) Western blot was employed for detecting the protein expression of p-JNK, LC3B, and p62 in VSMCs. (e, f) Image showing LC3B staining in each group of VSMCs infected with mRFP-GFP-LC3 adenovirus for 6 h. (g, h) Image showing the number of autophagosomes and autolysosomes in each group of VSMCs detected by transmission electron microscopy (red arrow: autolysosomes; white arrow: autophagosomes). Data are expressed as the mean ± SEM of at least three independent experiments. ^∗^ refers to *P* < 0.05; ^∗∗^ refers to *P* < 0.01.

The article "Activation of CD137 Signaling Enhances Vascular Calcification through c-Jun N-Terminal Kinase-Dependent Disruption of Autophagic Flux" was retracted in 2022. Reason: duplicated images.

**Figure 5:** Autophagosome-containing vesicles secreted by VSMCs stimulated by CD137 signaling could result in calcification. (a) Autophagosome-containing vesicle in agonist-CD137 group was collected and flow cytometry was used to detect the expression of LC3B of the vesicle. (b) Image showing the protein expression of LC3B in autophagosome-containing vesicle collected in each group. (c) BCA protein assay evaluated the concentration of autophagosome-containing vesicle secreted by VSMCs of each group. (d) VSMCs were cultured with PBS and agonist-CD137 group originated autophagosome-containing vesicle. Von Kossa staining was applied to indicate the calcification, and the expression of BMP2 in treated VSMCs was detected by immunohistochemistry. (e) Western blot was used to detect calcification markers of VSMCs extracted lysis. Data are expressed as the mean ± SEM of three independent experiments. ^∗^ refers to *P* < 0.05; ^∗∗^ refers to *P* < 0.01.

## Data Availability

The data used to support the findings of this study are available from the corresponding author upon request.
